The article "A security technology of power relay using edge computing" was retracted in 2024. Reason: concerns about the peer review.

# A security technology of power relay using edge computing

**DOI:** 10.1371/journal.pone.0253428

**Published:** 2021-09-02

**Authors:** Zhongqing Sang, Kai Yang, Rencheng Zhang

**Affiliations:** Key Laboratory of Process Monitoring and System Optimization for Mechanical and Electrical Equipment (Huaqiao University), Fujian Province University, Xiamen City, China; Ministry of Natural Resources North Sea Bureau, CHINA

## Abstract

The purposes are to find the techniques suitable for the safety relay protection of intelligent substations and discuss the applicability of edge computing in relay protection. Regarding relay protection in intelligent substations, edge computing and optimized simulated annealing algorithm (OSAA) are combined innovatively to form an edge computing strategy. On this basis, an edge computing model is proposed based on relay fault traveling waves. Under different computing shunt tasks, OSAA can converge after about 1,100 iterations, and its computing time is relatively short. As the global optimal time delay reaches 0.5295, the corresponding computing time is 456.27s, apparently better than the linear search method. The proposed model can reduce the computing time significantly, playing an active role in the safe shunting of power relays. The simulation also finds that the voltage and current waveforms corresponding to the fault state of Phase A are consistent with the actual situations. To sum up, this model provides a reference for improving and optimizing intelligent substation relay protection.

## Introduction

The continuous evolution of modern technologies and smart grid systems has put forward higher network demands than ever. The frequent security accidents in power grids also demand improved power network security and stability [1–3]. Relay protection is an important defense technique for smart grid systems; its device can alarm while clearing the faults so that the maintenance personnel can quickly identify the fault and take corresponding countermeasures [4]. As the power grid scale and security demand expand, higher requirements are set forth for power relay security protection. Furthermore, as edge computing displays excellent performance in intelligent applications, data optimization, and security assurance, it is applicable in power relay protection. In short, relay protection plays a pivotal role in improving the security performance of power networks [5, 6]. Edge computing has made power grid informatization and intelligent transformation possible, and its uniqueness has given it a wide application range. The essence of intelligent automation lies in the centralized processing based on control, during which computing tasks are completed according to the actual conditions of the signals [7, 8]. Edge computing is formed based on the comprehensive integration of the Internet of Things (IoT) and high bandwidth. Depending on the platform, edge computing can achieve signal control by providing low-latency data processing. Since edge computing can ensure security, optimize data, and protect privacy, it has an extensive applicability range in power grid systems [9, 10]. Regarding relay protection, the power relay protector can avoid many problems; however, if the device has performance problems, the power grid system’s security will be prone to hidden dangers.

The article "A security technology of power relay using edge computing" was retracted in 2024. Reason: concerns about the peer review.

At present, edge computing has been universally accepted in smart grids. However, the research on applying edge computing to relay protection is relatively scarce. Combining edge computing and relay protection optimization is bound to find a useful approach to protect power grid security. Thus, this study explores intelligent substations, optimizes the simulated annealing algorithm, and proposes a safe computing shunt strategy to seek technology of protecting power relay security. Based on the grid fault analysis, an edge computing model is constructed according to the relay-fault traveling waves to provide references for enhancing the security protection performance of intelligent grid systems.

## Literature research

### Research on edge computing applications in power grids

To date, the application of edge computing in the power grid has been extensively examined. Wang et al. (2020) introduced a blockchain mutual authentication and key negotiation protocol into the low-latency and real-time service in an intelligent grid’s operation based on edge computing. The protocol attained reasonable security guarantees in the security analysis and demonstrated excellent application potential in intelligent grid deployment [11]. Shrestha and Lin proposed a data-centric edge computing infrastructure, analyzing the hosting and defense mechanism in IoT by integrating the physical state of the dispersed grid area [12]. Ibrahim et al. (2020) reviewed the application of machine learning technology in intelligent grids and accentuated advanced computing and communication technologies’ prospects in intelligent grids, including edge computing, the IoT, and 5G wireless networks. Meanwhile, intelligent grids’ development trend of automation and intelligence was revealed [13]. Liu et al. (2020) explored the joint problem of rapid selection of charging stations and electric vehicle path planning and proposed a low-battery electric vehicle charging strategy based on deep reinforcement learning, using the software-defined network and e-vehicle edge computing technology. Reportedly, the intelligent grid system transmitted electricity using a two-way flow of electricity and information [14].

The article "A security technology of power relay using edge computing" was retracted in 2024. Reason: concerns about the peer review.

### Research on relay protection

There are currently countless works about relay protection. Suliman and Ghazal (2020) researched applications of field programmable analog arrays in designing and implementing overcurrent relays for power relay optimization. Based on MATLAB, they introduced the modeling and simulation methods of the protection system and provided actual test results for different faults. Results found that relay protection could quickly respond to steady-state faults, distinguish the fault states, and isolate the faulty section without affecting other networks [15]. Abdel-Salam et al. (2017) proposed a multifunctional digital relay. By analyzing and discussing its role in overcurrent, over-under-voltage, and over-under-frequency protection, this relay was found to be digital and small, with multiple protection functions [16]. Lee et al. (2019) introduced a 154kV single-phase superconducting fault current limiter system. Then, this system was applied to the actual power system based on a new protection algorithm. Results found that the algorithm could provide good performance in commercial relay protection [17]. Suo and Guo (2020) emphasized the importance of relay protection devices and power automation systems in the power equipment manufacturing industry. They introduced the thermal design process of the relay protection device processing equipment. Simulation analysis proved that thermal simulation could guide the structural design and optimize the structure, making the stand-alone structure more reasonable and achieving more effective heat dissipation [18].

The studies mentioned above indicated that edge computing technology had achieved fruitful results in the field of smart grids, involving a broad range of applications such as network data deployment, network defense mechanisms, and power supply. Edge computing exhibits excellent performance in these areas and provides many benefits for the further optimization and development of smart grids. However, despite the applications of edge computing in smart grids, research on relay protection and security protection using edge computing technology has been rarely reported.

The Methods section sequentially introduces smart substations and relay protection, the safety computing shunt strategy based on edge computing, and the edge computing model based on relay-fault traveling waves. The Results and Discussion section analyzes and characterizes the performance of the proposed optimized simulated annealing algorithm (OSAA) and the security performance requirements of power relay protection and fault traveling wave simulation results. The Conclusions section summarizes the research work and highlights the limitations and future research directions.

The article "A security technology of power relay using edge computing" was retracted in 2024. Reason: concerns about the peer review.

The contributions of this study are as follows: (i) a safety computing shunt strategy is proposed on the basis of edge computing and OSAA, providing a method for the safe shunt of power relays. The algorithm has good convergence performance and global optimal computing time. The delay computing time is markedly better than the linear search method. (ii) An edge computing model based on the relay-fault traveling wave is proposed. The model’s simulation results corroborate the actual situation in detecting current and voltage, providing an effective strategy for the optimization and promotion of power relay protection.

## Methods

Fig 1 summarizes the overall research process. Based on the analysis and explanation of intelligent substation and relay protection, edge computing is introduced; combined with OSAA, an edge computing strategy including computing task shunting, safety overflow probability, and resource allocation is proposed, as well as an edge computing model based on traveling waves of relay faults. By comparing the linear search method, the convergence performance and computing time of OSAA are analyzed; the requirements for the security performance of power relay protection are analyzed as well. The effectiveness of the power relay system is revealed by analyzing the fault traveling wave simulation results.

**Fig 1:** The overall research process.

### Intelligent substations and relay protection

An intelligent substation develops along with intelligent grids in the power grid system. Unlike conventional substations, intelligent substations incorporate intelligent devices, which are advanced, reliable, low-carbon, and environment-friendly. Functions like information collection, information measurement, protection, and monitoring can be automatically realized at intelligent substations [19, 20]. The intelligent substation equipment can be categorized into the following three types: station control layer, bay layer, and process layer. An intelligent terminal is an indispensable device in the process layer, connecting the primary and secondary equipment in the intelligent substation. The intelligent terminal’s functions regulate the switch circuit breaker, receiving the protection device’s trip command and communication. The intelligent substations’ intelligence embodies sensing and measuring technology, intelligent decision-making, and fault self-repair. Contrasting conventional substations’ equipment composition, electronic transformers, intelligent terminals, and merging units are introduced into intelligent substations. As vital secondary equipment, intelligent terminals are primarily accountable for protection, measurement, and control. Several new equipment introductions render the protection for electrical systems more effective in intelligent substations. Fig 2 shows the relay protection system’s composition in intelligent substations.

The article "A security technology of power relay using edge computing" was retracted in 2024. Reason: concerns about the peer review.

**Fig 2:** The relay protection system’s composition in an intelligent substation.

The relay protection structure has evolved rapidly with the quick development of intelligent substations. The network development of protection devices has become the focus of intelligent relay protection. Of note, relay protection is a vital system in intelligent substations. Unlike conventional substations, the relay protection system in intelligent substations primarily comprises three modules—information collection, operation decision-making, and decision execution [21, 22]. Besides, the merging unit and its electronic sensors collect relevant information in the intelligent substation, implying that signal collection in the intelligent substation no longer depends on the protection device.

Meanwhile, the intelligent terminal replaces the switch circuit breaker. Optical-fiber Ethernet transmission methods are extensively used in intelligent substations, enabling easy information-sharing, equipment operation, and maintenance. Compared with conventional substations, the relay protection’s advantages in intelligent substations lie in information-sharing realization, accessible new functions, communication networks’ usage, signal transmission’s reliability, electronic sensors’ application, easy device interoperability, and significant automation enhancement.

### A safe computing shunt strategy based on edge computing

Devices’ communication is highly problematic in the network transmission of intelligent substations, and security requirements and energy consumption limits vary for different intelligent terminals, resulting in significant differences in the data distribution strategy for different computing tasks. The resource allocation in the power network system often comprises multiple computing members, rendering resource allocation more challenging. The difference in security overflow probability affects the entire intelligent terminal’s computing delay and the shunt strategy [23], which is unfavorable for relay protection in intelligent substations. In this study, we proposed a safe computing shunt strategy for the equipment’s energy and security requirements based on edge computing and two edge computing servers for intelligent terminals in power relay protection. Fig 3 presents the data transmission scenario, which has two edge computing servers and one intelligent terminal.

The article "A security technology of power relay using edge computing" was retracted in 2024. Reason: concerns about the peer review.

**Fig 3:** Data transmission scenario.

Eqs (1) and (2) show the transmission power acquired by calculating the intelligent terminal’s shunt based on two edge servers.

$$p_{iT}^{1}=\frac{n_{p}2^{\frac{s_{i}^{up,1}}{t_{i}^{up,1}W_{T}(1-\varepsilon_{iT}^{1})}}-n_{p}}{{\hat{g}}_{iT}^{1}-\theta_{iT}^{1}2^{{}^{\frac{s_{i}^{up,1}}{t_{i}^{up,1}W_{T}(1-\varepsilon_{iT}^{1})}}}}$$ (1)

$$p_{iT}^{2}=\frac{n_{p}2^{\frac{s_{i}^{up,2}}{t_{i}^{up,2}W_{T}(1-\varepsilon_{iT}^{2})}}-n_{p}}{{\hat{g}}_{iT}^{2}-\theta_{iT}^{2}2^{{}^{\frac{s_{i}^{up,2}}{t_{i}^{up,2}W_{T}(1-\varepsilon_{iT}^{2})}}}}$$ (2)

where $p_{iT}^{1}$ denotes the first edge computing server’s transmission power; $p_{iT}^{2}$ denotes the second edge computing server’s transmission power; $s_{i}^{up,1}$ and $s_{i}^{up,2}$ denote the two edge computing servers’ optimal upload workload, respectively; *W*_*T*_ depicts the server bandwidth; *n*_*p*_ denotes the background noise power; $t_{i}^{up,1}$ and $t_{i}^{up,2}$ signify the transmission time from the intelligent terminal to the servers 1 and 2, respectively; $\varepsilon_{iT}^{1}$ and $\varepsilon_{iT}^{2}$ represent the security overflow probability from the intelligent terminal to the servers 1 and 2, respectively; ${\hat{g}}_{iT}^{1}$ and ${\hat{g}}_{iT}^{2}$ denote the channel gains from the intelligent terminal to the two edge computing servers, respectively; and $\theta_{iT}^{1}$ and $\theta_{iT}^{2}$ represent the two parameters associated with the two edge computing servers’ security overflow probability, respectively.

The computing result attained from the intelligent terminal returned through the edge server. Eqs (3) and (4) present the downlink transmission power:

$$p_{Ti}^{1}=\frac{n_{p}2^{\frac{s_{i}^{do,1}}{t_{i}^{do,1}W_{T}(1-\varepsilon_{Ti}^{1})}}-n_{p}}{{\hat{g}}_{Ti}^{1}-\theta_{Ti}^{1}2^{{}^{\frac{s_{i}^{do,1}}{t_{i}^{do,1}W_{T}(1-\varepsilon_{Ti}^{1})}}}}$$ (3)

$$p_{Ti}^{2}=\frac{n_{p}2^{\frac{s_{i}^{do,2}}{t_{i}^{do,2}W_{T}(1-\varepsilon_{Ti}^{2})}}-n_{p}}{{\hat{g}}_{Ti}^{2}-\theta_{Ti}^{2}2^{{}^{\frac{s_{i}^{do,2}}{t_{i}^{do,2}W_{T}(1-\varepsilon_{Ti}^{2})}}}}$$ (4)

where $p_{Ti}^{1}$ denotes the first edge computing server’s downlink transmission power; $p_{Ti}^{2}$ signifies the second edge computing server’s downlink transmission power; $s_{i}^{do,1}$ and $s_{i}^{do,2}$ denote the two edge computing servers’ optimal transmission power of downlink transmission workloads, respectively; $t_{i}^{do,1}$ and $t_{i}^{do,2}$ denote the optimal downlink transmission time from the intelligent terminal to the servers 1 and 2, respectively; $\varepsilon_{Ti}^{1}$ and $\varepsilon_{Ti}^{2}$ denote the security overflow probability from servers 1 and 2 to the intelligent terminal; ${\hat{g}}_{Ti}^{1}$ and ${\hat{g}}_{Ti}^{2}$ denote the channel gains from the two edge computing servers to the intelligent terminal, respectively; and $\theta_{iT}^{1}$ and $\theta_{iT}^{2}$ signify the two parameters associated with the two edge computing servers’ security overflow probability, respectively.

The article "A security technology of power relay using edge computing" was retracted in 2024. Reason: concerns about the peer review.

The safe computing shunt strategy proposed in this study comprises the optimization of computing task shunting, security overflow probability, and resource allocation to realize the computing tasks’ comprehensive delay by the intelligent terminals’ minimization. Eq (5) shows the realization based on the calculated date quantity $s_{i}^{up,1}$ and $s_{i}^{up,2}$ shunted to server 1 by the intelligent terminal and the upload time’s minimization in server 1 by energy distribution factor *α*.

$$t_{i(s_{i}^{up,1},s_{i}^{up,2},\alpha )}^{up,1*}=\min t_{i}^{up,1}$$ (5)

where $t_{i(s_{i}^{up,1},s_{i}^{up,2}.\alpha )}^{up,1*}$ denotes the optimal local solution.

Eq (6) presents the realization based on the calculated date quantity $s_{i}^{up,1}$ and $s_{i}^{up,2}$ shunted to server 1 by the intelligent terminal and the upload time’s minimization in server 2.


$$t_{i(s_{i}^{up,1},s_{i}^{up,2},\alpha )}^{up,2*}=\min t_{i}^{up,2}$$ (6)

Accordingly, Eq (7) presents the transmission delay’s local optimal solution returned to the intelligent terminal after evaluating the edge server 1.


$$t_{i(s_{i}^{up,1},s_{i}^{up,2},\alpha )}^{do,1*}=\min t_{i}^{do,1}$$ (7)

Eq (8) presents the transmission delay’s local optimal solution for edge server 2.


$$t_{i(s_{i}^{up,1},s_{i}^{up,2},\alpha )}^{do,2*}=\min t_{i}^{do,2}$$ (8)

Eq (9) demonstrates that edge server 1’s computing and transmission time summation for the top-level problem is set after converting the bottom-level problem.


$$t_{i(s_{i}^{up,1},s_{i}^{up,2},\alpha )}^{temp,1*}=t_{i(s_{i}^{up,1},s_{i}^{up,2},\alpha )}^{up,1*}+t_{i(s_{i}^{up,1},s_{i}^{up,2},\alpha )}^{do,1*}+\frac{s_{i}^{up,1}}{V^{ser,1}}$$ (9)

Likewise, Eq (10) shows edge server 2’s computing and transmission time summation for the top-level problem.


$$t_{i(s_{i}^{up,1},s_{i}^{up,2},\alpha )}^{temp,2*}=t_{i(s_{i}^{up,1},s_{i}^{up,2},\alpha )}^{up,2*}+t_{i(s_{i}^{up,1},s_{i}^{up,2},\alpha )}^{do,2*}+\frac{s_{i}^{up,2}}{V^{ser,2}}$$ (10)

In Eqs (9) and (10), *V*^*ser*,1^ and *V*^*ser*,2^ denote the computing speeds of edge computing servers 1 and 2, respectively.

With the given $s_{i}^{up,1}$ and $s_{i}^{up,2}$, Eq (11) presents the optimal local delay $t_{i(s_{i}^{up,1},s_{i}^{up,2})}^{ove*}$.


$$t_{i(s_{i}^{up,1},s_{i}^{up,2})}^{ove*}=\min\;\max\{t_{i(s_{i}^{up,1},s_{i}^{up,2})}^{loc},t_{i(s_{i}^{up,1},s_{i}^{up,2})}^{temp,1*},t_{i(s_{i}^{up,1},s_{i}^{up,2})}^{temp,2*}\}$$ (11)

In this study, we adopted the simulated annealing algorithm to solve the top-level problem [24, 25]; this algorithm was optimized and defined as OSAA. First, the initial temperature, descending temperature, minimum temperature, and annealing times were initialized, and a set of initial solutions were randomly generated and expressed as $\left[s_{i}^{up,1},s_{i}^{up,2}\right]$. After solving the optimal local solution, the previous underlying processing method was used to solve the optimal local solution with $\left[s_{i}^{up,temp1},s_{i}^{up,temp2}\right]$ given. Then, we calculated and compared the difference between the optimal solution before and after the update processing. If the difference was <0, the sum of $t_{i(s_{i}^{up,temp1},s_{i}^{up,temp2})}^{ove*}$ and $\left[s_{i}^{up,temp1},s_{i}^{up,temp2}\right]$ was updated, and a random number distributed uniformly within (0,1) was generated. After $t_{i(s_{i}^{up,temp1},s_{i}^{up,temp2})}^{ove*}$ and $\left[s_{i}^{up,temp1},s_{i}^{up,temp2}\right]$ were further updated, the top-level problem’s optimal solution sum $t_{i(s_{i}^{up,temp1},s_{i}^{up,temp2})}^{ove*}$ and $\left[s_{i}^{up,temp1},s_{i}^{up,temp2}\right]$ were output finally. On this basis, the implementation process of OSAA is displayed in Fig 4 below.

The article "A security technology of power relay using edge computing" was retracted in 2024. Reason: concerns about the peer review.

**Fig 4:** Implementation process of OSAA.

To test the proposed algorithm, the scenario composition parameters are set as follows: (1) the edge server 1 is at (300m, 0m), (2) the edge server 2 is at (-300m, 0m), (3) the smart terminal is at the origin, and (4) the radius is 300m. Moreover, the background noise power is set to 10^**−8**^, the computing speed of the corresponding smart terminal is set to 10Mbps, the upper limit of the energy consumption is 3.5J, the corresponding compression ratio is 0.35, and the computing power consumption of the server is set to 0.2. Different initial computing shunt tasks were set to test the proposed OSAA’s efficacy and convergence. Besides, a linear search method was introduced to validate the algorithm’s performance and its applicability in the power relay protection system’s intelligent terminal at different edge server processing speeds by comparing and analyzing the two algorithms’ simulation results.

### Edge computing model using relay-fault traveling wave

The development of edge computing corroborates the intellectual development of power grids. Fig 5 shows an edge computing-based relay protection system for the delayed and real-time traditional power grid relay protection [26, 27]. In this system, the critical data are transmitted to the edge device by the relay protection equipment and its intelligent terminals. After authenticating the related access terminal, it obtained feedback by the protocol analysis and transmitted the prediction results and related suggestions based on the data to the background system. Unlike conventional relay systems, access to the electric power private cloud in edge computing can extract data and attain more simulation and prediction results.

The article "A security technology of power relay using edge computing" was retracted in 2024. Reason: concerns about the peer review.

**Fig 5:** Relay protection system in edge computing.

Relay protection devices realize electrical protection based on power-frequency electrical quantity in the power network, guaranteeing the entire system’s stable operation [28]. Nevertheless, based on the power-frequency electrical quantity, some protection problems persist in the application, including trouble providing complete guarantee measurement accuracy, small fault current and inadequate characteristics in selecting the line connection, and unsmooth system operation with unstable currents. Compared with this traditional protection method, the protection equipment based on the traveling electrical wave quantity is unaffected by system oscillation and long-line distributed capacitance. Conceptually, traveling waves depict the propagated voltage and current electromagnetic waves along the transmission line. The superposition principle can analyze the faults in the line. With the traveling waves’ protection, the load component of the average state is not displayed; thus, the component discussion can separately perform the fault analysis. We constructed a loop circuit network for the fault traveling waves’ simulation analysis in power relays on the MATLAB simulation platform. The loop circuit comprised three power supplies and four distributed parameter transmission lines; the three-phase power supply was adopted in the power supply model [29, 30]. Table 1 lists the three power supplies’ parameter settings.

**Table 1:** The three power supplies’ parameter settings.

Parameter	Set value	Parameter	Set value
Phase-to-phase voltage (Vrms)	524e3	Power supply resistance (Ohms)	5.75
Angle of phase A (degrees)	0	Power supply inductance (H)	0.0453
Frequency (Hz)	50	Base voltage (Vrms ph-ph)	0

For the distributed parameter transmission lines, the lengths in lines 1–2, 2–3, and 3–4 were 100, 150, and 250 km, respectively. In the power relay simulation model, the measurement module’s role based on the three-phase power supply was to transmit the relevant current and voltage signals acquired by detecting the oscilloscope. The “To File” module realized the documents’ format conversion and storage. After the simulation of the power relay circuit fault based on the simulation model mentioned above, the forward and reverse traveling wave extraction could be realized according to the faults in the relevant data. Fig 6 shows the extraction process.

The article "A security technology of power relay using edge computing" was retracted in 2024. Reason: concerns about the peer review.

**Fig 6:** Fault traveling wave’s extraction process.

In the power relay’s simulation analysis, the detection duration in the test was 0.10 s. For the faults in the three-phase line, phase A was assumed to be short-circuited.

## Results and discussion

### The OSAA performance analysis

Fig 7(A) and 7(B) shows the proposed OSAA’s convergence with 1600 iterations in different computing offload tasks.

**Fig 7:** OSAA’s convergence in different computing offload tasks: (a) $s_{i}^{up,1}=10Mbits,s_{i}^{up,2}=10Mbits$; (b) $s_{i}^{up,1}=8Mbits,s_{i}^{up,2}=12Mbits$.

The global convergence delay corresponding to the final convergence state remained the same even when the safe computing shunt’s uploading tasks differed. The global optimal delay had a minimum value with the iterations number approximately 1100, suggesting the OSAA reaches convergence after about 1100 iterations. Chen et al. (2020) proposed a hybrid relay for computing offloading problems. This relay reduced power consumption and time delay by jointly optimizing the computing-offloading ratio, bandwidth allocation, processor speed, and transmission power. It was also an iterative algorithm that significantly reduced the computing complexity [31]. The proposed model also shows good convergence. To test the superiority of OSAA further, it is compared with the linear search method.

With the edge server’s processing speed of 15 and 30 Mbps and the intelligent terminal’s computing demand in the power relay protection system 10–40 Mbit, the optimized algorithm was simulated. Fig 8 shows the OSAA’s simulation results in the global optimal computing delay and computing time based on the edge computing model of the relay-fault traveling wave.

**Fig 8:** Computing time simulation results of the OSAA and linear search method. GOD, the global optimal time delay; LS, the linear search method; and T, the computing time.

The analysis of the two algorithms’ global optimal computing delay and computing time indicated that with the same global optimal computing delay, the OSAA’s computing time was markedly less than the linear search method. For example, with a processing speed of 15 Mbps and a global optimal computing delay of 0.5295, the OSAA’s computing time was 456.27 s, whereas that with the linear search method was 2510.46 s. With a processing speed of 30 Mbps and a global optimal computing delay of 0.4881, the OSAA’s computing time was 462.25 s, whereas that with the linear search method was 3109.23 s. The OSAA reduced the computing time markedly and performed better than the linear search method in computing time. Furthermore, the above-described analysis of the algorithm convergence and the global optimal computing delay revealed that the proposed OSAA had applicability in the safe power relays shunting.

The article "A security technology of power relay using edge computing" was retracted in 2024. Reason: concerns about the peer review.

The reason may be the introduction of OSAA to the proposed model so that the solution to the top-level problem can be accelerated. On this basis, the final optimal solution based on the top-level problem can be output faster by determining the local optimal solution. Once the amount of tasks uploaded in edge computing is different, the minimum global optimal delay value can be obtained after some iterations; thus, the convergence performance of the algorithm is improved, and the computing time is also shortened. Regarding the relay protection of the power grid, faults can be discovered quickly, thereby improving problem-solving efficiency. Gusev et al. (2019) analyzed an unbiased edge computing scheme. They found that the distributed equipment-less data and computing offloading methods were energy-efficient, providing greater scalability and fault tolerance [32]. This scheme is similar to the proposed model; nevertheless, OSAA provides a wider application range and applicability.

### Analysis of the security performance requirements of the power relay protection

Fig 9 presents the impact of different eavesdropping channel strength on the optimal distribution scheme in edge computing servers 1 and 2 as the intelligent terminals’ security performance requirements in the power relay system change.

**Fig 9:** The impact of different eavesdropping channel strengths on the optimal distribution scheme. *β*, the eavesdropping channel strength.

Fig 9 suggests that when the upper limit of security overflow probability increases, that is, when the intelligent terminal in the power relay system has a relatively flat demand for security performance, the global optimal delay decreases, and the computing tasks of optimal computing shunting increases. Fig 10 shows the impact of the security overflow probability’s upper limit on the two edge computing servers’ optimal security overflow probabilities and the optimal transmission delays.

**Fig 10:** The impact of the security overflow probability’s upper limit on two edge computing servers’ optimal security overflow probabilities and optimal transmission delays.

Fig 10 demonstrates that the optimal upstream security overflow probabilities of edge computing servers 1 and 2 increase first and tend to be stable. Concurrently, as the security overflow probabilities’ upper limits increase, the two edge computing servers’ optimal transmission delays decrease.

The article "A security technology of power relay using edge computing" was retracted in 2024. Reason: concerns about the peer review.

Overall, the abovementioned change trend is that when the intelligent terminal’s requirements for security performance in the power relay system are lower, more workload can be uploaded to the edge computing server based on the computing shunt’s advantages. Thus, the optimal delay is reduced on the whole, and the uploading tasks’ workload increases. Meanwhile, when the security overflow probability’s upper limit increases, the intelligent terminal has more space to select the optimal security overflow probability. The impact of the security overflow probability’s upper limit on the optimal transmission delay revealed that transmission rates of intelligent terminals and edge computing servers were increasing. The proposed OSAA can briefly optimize the power relay system’s security performance and transmission delay with a limited energy budget, including intelligent terminals and edge computing servers in the power relay system. The two can reach a balance in particular conditions.

### Simulation results of the fault traveling waves

Fig 11(A)–11(C) shows the fault traveling waves’ simulation results in the power relay system based on edge computing.

**Fig 11:** The fault traveling waves’ simulation results in a power relay system based on edge computing: (a) voltage at detection point; (b) current at detection point; (c) forward and reverse traveling waves.

The waves in Fig 11 show that the detection point’s voltage and current waves after simulation align with the current and voltage characteristics when phase A is short-circuited, thereby validating the proposed simulation model’s efficacy and correctness. Moreover, phase A’s forward and reverse voltage traveling waves were consistent.

In the power relay system, the fault traveling waves’ effective extraction is significant for power faults analysis. We analyzed the characteristics of relay protection in the power system by modeling and simulation from fault traveling waves, offering a new direction and security development ideas to augment the security performance of relay protection. The simulation results based on the detection point’s voltage and current established the simulation model’s efficacy, providing a more intuitive understanding of the power relay’s operating characteristics. Nonetheless, an in-depth understanding of power system failures is significant for improving the power relays’ protection.

## Conclusions

An edge computing strategy is proposed. Comparing it with the linear search method reveals that OSAA provides excellent convergence performance while computing the top-level problems. If the global optimal computing delay is different, the computing time is reduced significantly, which is effective in the edge computing of power relay protection systems. Moreover, an edge computing model is proposed based on power relay fault traveling wave simulation. Results demonstrate that the voltage and current characteristics of Phase A in the fault state are consistent with changes in the actual situation. In short, the proposed safety computing shunt strategy based on edge computing consumes less time, and the OSAA displays good convergence performance. Meanwhile, the edge computing model based on relay-fault traveling waves can reflect the actual fault situation. The fault identification and analysis of relevant equipment is the key. The results can provide a feasible direction for the further improvement of power relay protection performance.

The article "A security technology of power relay using edge computing" was retracted in 2024. Reason: concerns about the peer review.

Smart grid is a very complex system. In the proposed edge computing strategy based on OSAA, only two edge computing servers and one smart terminal are considered. This is an ideal situation, which may be deviated from the actual situation. The fault traveling wave belongs to a module in the power relay protection; however, it does not yet represent the whole. Hence, future works will include more edge computing servers and smart terminals for analysis, and different details and levels that affect power relay protection will be discussed.

## Supporting information

S1 Data (RAR)
